# Optimization of College English Classroom Teaching Efficiency by Deep Learning SDD Algorithm

This article has been retracted.

**DOI:** 10.1155/2022/1014501

**Published:** 2022-01-21

**Authors:** Wei Zhang, Qian Xu

**Affiliations:** ^1^Department of Preschool Education, Hebei Women's Vocational College, Shijiazhuang 050000, China; ^2^Department of Economic Management, Hebei Women's Vocational College, Shijiazhuang 050000, China

## Abstract

In order to improve the teaching efficiency of English teachers in classroom teaching, the target detection algorithm in deep learning and the monitoring information from teachers are used, the target detection algorithm of deep learning Single Shot MultiBox Detector (SSD) is optimized, and the optimized Mobilenet-Single Shot MultiBox Detector (Mobilenet-SSD) is designed. After analyzing the Mobilenet-SSD algorithm, it is recognized that the algorithm has the shortcomings of large amount of basic network parameters and poor small target detection. The deficiencies are optimized in the following partThrough related experiments of student behaviour analysis, the average detection accuracy of the optimized algorithm reached 82.13%, and the detection speed reached 23.5 fps (frames per second). Through experiments, the algorithm has achieved 81.11% in detecting students' writing behaviour. This proves that the proposed algorithm has improved the accuracy of small target recognition without changing the operation speed of the traditional algorithm. The designed algorithm has more advantages in detection accuracy compared with previous detection algorithms. The optimized algorithm improves the detection efficiency of the algorithm, which is beneficial to provide modern technical support for English teachers to understand the learning status of students and has strong practical significance for improving the efficiency of English classroom teaching.

## 1. Introduction

At present, internationalization is in a stage of rapid development, and social enterprises have higher requirements for the English level of talent. Because college English teaching not only has the characteristics of the subject itself but also needs to meet the overall requirements of current quality education. The teaching of English in colleges and universities strives for the comprehensive development of students, which makes the structure of college English teaching very complicated, and it is difficult to guarantee teaching efficiency. With the change of educational concepts, the number of university classrooms is also showing a rapid increase. In the actual teaching process, the teacher needs to teach multiple students at the same time, and it is difficult to pay attention to all the students. The development of big data, using many monitoring resources in the classroom, combined with target detection in deep learning, provides research ideas for detecting student learning status and improving student teaching efficiency [1].

At present, many video target detections are derived from static image target detection. Zhao et al. studied that if the target detection model of the static image is directly used in the video target detection, the effect is very poor. Therefore, scholars combine the time and context information of the video to perform target detection [2]. Initially, the postprocessing stage completes the detection by a single frame of images. However, this method is mostly multistage, the results of each stage are affected by the results of the previous stage, and it is troublesome to correct errors in the previous stage. There are unclear problems caused by out-of-focus and object motion in the video, and this problem is not solved very well in the postprocessing stage [3]. Dou et al. [4] used optical flow, Long-Short Term Memory (LSTM), and Artificial Neural Network (ANN) to aggregate video time and context information to optimize the features of fuzzy frames, to make the detection accuracy better. In addition, the concept of key frames is introduced, the detection time is optimized, and optical flow-related technologies are used to give feature propagation. Recurrent Neural Networks (RNN) combined with lightweight and heavyweight feature extractors are interleaved and used to further improve the accuracy and speed of video target detection [5]. There are many shortcomings in the detection speed and accuracy of the current research compared with previous studies [6–9]. Affected by the detection target, its performance will also have a certain gap. Its availability in complex environments, dense target detection, and lightweight model design still needs great improvement [10].

The deep learning Single Shot MultiBox Detector (SSD) algorithm is optimized. Through the analysis of the algorithm, a series of improvements have been made to the deficiencies of its large amount of basic network parameters and poor detection of small targets. The SSD base network is reasonably replaced. The characteristics of the deep separable convolutional network are used to optimize the network parameters to enhance computational efficiency. The data in the deep feature map is merged upward in the shallow layer, and the accuracy of the calibration of small targets can be improved. Finally, experiments related to student behavioural state are analysed. This proves that the accuracy of small target recognition has been improved without changing the calculation speed of traditional algorithms. These help teachers understand the students' learning status and are of great significance to the improvement of English classroom teaching efficiency.

The structure is arranged as follows: Section 1 is the introduction, which introduces related research results in the detection field; Section 2 is the research method, which introduces the design process of the algorithm in detail; Section 3 is the experimental results, testing and analysing the performance of the designed algorithm; Section 4 is the conclusion, summarizing the research algorithm and explaining the future research direction.

## 2. Materials and Methods

### 2.1. Target Detection in Deep Learning

As a frequently used deep learning network, the neural network is composed of many neurons. It has two functions, linear and nonlinear functions in sequence. The output of the linear function is not related to the number of layers, and it is always linear, so the scope of application is limited [11]. However, reality is often very complicated, and the neural network needs to analyse and process many nonlinear problems, so a function is used to activate the result. Such a neural network can analyse and process nonlinear problems [12]. The calculation process of the activation function is shown in Figure 1.

In the activation function calculation process in Figure 1, the input is placed in the god cell, the neuron is linearly calculated on it and then transferred to the activation function, and the neuron can get a nonlinear result [13]. The application of the activation function in the neural network enhances its representation ability.

The Sigmoid function originally originated from the biological field, and it is also called the Logistic function. Its function image looks like the letter S, with an increasing trend in general. Its output is in the range of 0 and 1, so it is used on the output of the activation network layer [14]. The Sigmoid function is shown in equation (1):

(1) $$\begin{array}{c} f\left(z\right)=\frac{1}{1+e^{-z}}. \end{array}$$

In equation (1), *f*(*z*) represents the required loss function, and *z* is the input value. This function is generally used to solve two classifications. Although it has its own advantages, it can be handled well in some projects, but when using this method to obtain the derivative, the program will be more troublesome, and sometimes, there will be the problem of vanishing gradient [15].

The Rectified Linear Unit (ReLU) function is a linear rectification function. Image recognition and computer vision are widely used. Its function equation is

(2) $$\begin{array}{c} f\left(x\right)=\max\left(x,0\right). \end{array}$$

In the function equation, *f*(*x*) represents the function that requires the loss, and *x* is the input. The calculation of this function is relatively simple, so its calculation speed is excellent. In the calculation, some neurons are set to 0, so the network will be very sparse so that the problem of overfitting is optimized [16].

The Soft version of max (Softmax) function is also called the normalized exponential function. Its result is maintained at (0, 1), and the sum of the probability of satisfying the output result is 1, as shown in equation (3):

(3) $$\begin{array}{c} f{\left(x\right)}_{j}=\frac{e^{x_{j}}}{\sum_{k=1}^{k}e^{x_{j}}},\;\left(j=1,\ldots ,k\right). \end{array}$$

In equation (3), *f*(*x*)_*j*_ is the value of the loss function, *x*_*j*_ is the *j*-th input, and *k* is the number of input values. The function works well on multiclassification problems; however, the isolation effect between different categories is slightly insufficient [17].

### 2.2. Convolutional Neural Network (CNN) Structure

As the basis for exploring deep learning, Convolutional Neural Network (CNN) has a network structure divided into three layers: input data, output data, and intermediate layer [18]. The specific CNN structure is shown in Figure 2.

In the CNN structure, the input layer can analyse multidimensional data. When inputting relevant data into the network, it is necessary to unify the time and frequency of the relevant data. The output layer is to output the corresponding results of specific problems and classify the problems. The output is related to the object category. In the positioning problem, the output is the coordinate data of the object. The middle layer is divided into three layers: convolutional layer, pooling layer, and fully connected layer, which will be introduced one by one in the following [19].

The most important part of the convolutional layer is the convolution kernel. The convolution kernel can also be regarded as a matrix of elements, and different elements will have corresponding weights and bias coefficients. When performing a convolution operation, the input data will be scanned with a certain rule. The function of the pooling layer is to delete invalid information in the data obtained by the upper layer and reduce the size. Generally, there are average pooling, maximum pooling, overlapping pooling, and maximum pooling. The first and second types are widely used. The function of the fully connected layer is used to classify the information data from the previous layer. In special cases, the previous operation can be replaced with the average value of the entire parameter value, which can reduce the target of redundant data [20].

CNN generally has the following two characteristics:

1. Local area connection. Normally, neurons are connected to each other when the network is connected. In CNN, it is only partially connected. If there are connections between *N*−1 layers of neurons and *N* layers of neurons, the connection form of CNN is shown in Figure 3.
2. Weight sharing. The convolution kernel of the convolutional layer can be regarded as an element matrix, and the convolution operation is to use the convolution kernel to scan the information. For example, if a 3*∗*3*∗*1 convolution kernel has 9 parameters, input an image to pass this convolution. The integration kernel performs related convolution processing, and the entire image will share these 9 parameters during scanning.

### 2.3. Methods of Face Recognition and Image Preprocessing

In face recognition, multitask convolutional neural (MTCNN) face detection algorithm, affine transformation face alignment, and Insightface face comparison algorithm are analysed. When performing student face recognition, the process shown in Figure 4 is used for recognition and detection.

In the face recognition process in Figure 4, the relevant face data set should be prepared, and then the MTCNN algorithm is used to align the face with the affine transformation. The processed data is processed in Insightface for information comparison, and finally, the recognition result is obtained. The entire recognition process is over. In the algorithm selected in this paper, the MTCNN face detection model uses the image pyramid multiscale face detection method as the basis and uses its subnetwork to obtain the relevant features of the face in order to lay the foundation for correcting the direction of the face. When correcting the face, the method of affine transformation is used to align the face. Since the face images do not always show a very regular face, the change of the angle will have a great influence on the recognition, and it is more important to correct the face. Through the above MTCNN face detection algorithm, the key points of the face are obtained as a basis, and appropriate changes such as translation, rotation, and scaling are used to achieve the purpose of face alignment. The geometric transformation of the image is realized by the affine transformation method. The combination of translation-related image transformation is affine transformation, which uses the linear change from two-dimensional coordinates to achieve the mapping between the image and the image, and the flatness and parallelism of the image do not change during this process. The Insightface face comparison method used in face recognition reduces the distance within the class so that the class is closer, and many features with angular characteristics are obtained so that the performance of the face recognition model is enhanced.

Under normal circumstances, the image has many interferences such as a lot of noise, and the information effect will be affected to varying degrees. In order to ensure that the quality of the image to be operated meets the standard, the preprocessing of the image is necessary. As shown in Figure 5, several common image processing methods are used.

In Figure 5, normalization is to transform the image into a standard mode, use the image invariant moments to find a set of parameters, and use it to reduce the interference of other functions on the image. Its essence is to find the amount of the image that does not change. After the shape brightness operation is performed on it, the changed image and the original image can be classified into one category.

### 2.4. Classroom Behaviour Recognition Model Design Process

As far as classroom teachers are concerned, mastering the relevant behaviours of students in the classroom can obtain the current state of the students in class and then make corresponding adjustments to improve teaching efficiency. Combining the relevant characteristics of students' behaviour in the classroom, an optimized SSD algorithm is designed [21]. The specific recognition process of the constructed classroom behaviour recognition model is shown in Figure 6.

Specifically, the application of the behaviour recognition process in the classroom is mainly by the following aspects:

1. Collect student behaviour images. Find enough images of behaviours such as raising hand, sitting upright, writing, sleeping, and playing with mobile phone in class. The number of each action is equal.
2. Build an identification database. The collected images are preprocessed and labelled, and the images are divided into training set, test set, and verification set according to the proportions.
3. Train and test the model. Let the training set be trained in the behaviour recognition network model to obtain the initial model, test the model through the validation set, and then adjust the network model parameters according to the results. Use the test data in the model to observe whether the output results meet the expectations, to decide whether to continue training or not, retain the behaviour recognition model with excellent recognition effect, and use it in the subsequent classroom behaviour recognition [22].

### 2.5. Optimization Design of SSD Target Detection Algorithm

The target detection algorithm is an improvement and optimization on SSD, so it is necessary to understand the structure of the original algorithm model and the principle of prioritization [23]. According to the input image size, it can be divided into SSD300 and SSD512. SSD300 is used. Its network structure is divided into two parts. One is the main part of the network, also known as the basic network. It comes from the relevant subtype network. The second is the convolutional network added later. Its function is to assist the previous network in acquiring image features more deeply [24]. Delete the fully connected layer behind Visual Geometry Group Network 16 (VGG16), and keep the previous part of the convolutional network. Use the two newly created convolutional layers in the deleted places, named Convolution 6 (Conv6) and Conv7, add eight slowly decreasing convolutional layers to the end, and then add the classification layer and the nonmaximum suppression layer. The SSD network structure is shown in Figure 7.

SSD is a one-stage target detection algorithm [25]. In the process of feature extraction, the SSD algorithm uses multiscale feature maps for detection, adds a gradually decreasing convolution layer to the modified VGG16 network, and then selects 6 layers from all levels for prediction. They are Conv4_3, Conv7, Conv8_2, Conv9_2, Conv10_2, and Conv11_2, and the size is slow to take effect from front to back. In the feature map, the relatively large size is used to identify small objects, and the smaller one is used to identify large objects [26]. In this way, image features can be obtained at different levels, and not only can shallow-level data information be obtained, but also deeper-level information can be obtained.

The goal of basic network improvement is to replace the original backbone network VGG16 with a lightweight network. By consulting relevant information, the Mobilenet network is more suitable for the requirements here because it uses depth separable convolution to replace ordinary convolution to reduce the number of parameters. Compared with the hundreds of millions of parameters in VGG16, the Mobilenet network only contains 4.2 million parameters. Therefore, Mobilenet is used as the foundation, and after certain improvements, it is used as the basic network of SSD [27].

The following is an introduction to specific Mobilenet improvements. The related situation of basic improvement is shown in Figure 8.

(1) Mobilenet has been improved. Mobilenet is more efficient than VGG16, mainly manifested in the following: (1) depthwise separable convolution is used to construct the network; (2) width coefficient and resolution coefficient are used. It uses two parts to complete a convolution operation, followed by deep convolution and point convolution [28]. If they are regarded as two layers, then the Mobilenet network structure has a total of 28 layers. On the contrary, if they are regarded as one layer, then there are 14 layers. The essence of the depth separable convolution is to perform the convolution operation in two steps. When the image is transferred to the network, it is necessary to use the deep convolution operation to obtain the relevant feature information data and perform the Batch Normalization (BN) and Rectified Linear Unit (ReLU) operations on the previously obtained feature maps. Then use the point convolution operation to obtain other pieces of relevant feature map information. After that, BN and ReLU are used here to get the following results. The ratio of the depth separable convolution and the standard convolution parameter can be obtained by equation (4):
  (4) $$\begin{array}{c} \frac{F_{k}*F_{k}*F_{f}*F_{f}*R+1*1*F_{f}*F_{f}*R*P}{F_{k}*F_{k}*R*P*F_{f}*F_{f}}=\frac{P+F_{k}^{2}}{PF_{k}^{2}}. \end{array}$$
In equation (4), *F*_*k*_ is the value of the convolution kernel and the size of the *F*_*f*_ shi image.
In order to reduce the network parameters, it is necessary to use not only the depth separable convolution but also the width coefficient *a* and the resolution coefficient *ρ*. More values for *a* are 1, 0.75, 0.5, and 0.25. The function of *a* is to reduce the number of channels. For example, an input channel with a value of *R* is converted into *αR* after being added, and the amount of calculation is reduced. The reduced value is *α*^2^. The amount of calculation is also affected by the resolution, so the function of *ρ* is to reduce the object resolution. After they are used, the calculation amount of the pixel value is reduced by *ρ*^2^. The above is the related improvement measures taken for Mobilenet.
When performing model training and learning, it is necessary to continuously observe the change of the loss function. When the value of the loss function continues to decrease, it means that the result of model training is approaching the best result. During the gradient descent, the amplitude of the value swing may become extremely large or not change, making the gradient descent speed slower. So, the addition of optimization algorithms is obviously very important. Root Mean Square Prop (RMSProp) optimization algorithm is used. This algorithm obtains the historical gradients of all dimensions and squares them. After superposition, the attenuation rate is added to obtain the relevant historical gradient sum. In the parameter update process, the learning rate is divided by the value calculated by equation (4). After using this optimization algorithm, the gradient direction is maintained within a small range, and the network convergence speed is well optimized. Its specific calculation is as equation (5):
  (5) $$\begin{array}{c} S_{sR}=\beta S_{\text{d}R}+\left(1-\beta \right){\left(\text{d}R\right)}^{2}, \end{array}$$
  (6) $$\begin{array}{c} R=R-\rho \frac{\text{d}R}{\sqrt{S_{\text{d}R}+a}}. \end{array}$$
In equations (5) and (6), *β* is the decay rate. *S*_*R*_ is the cumulative gradient variable. *ρ* is the learning rate. *a* is a constant, and its function is to avoid the situation where the denominator is 0. *R* is the parameter.
(2) Replacement of SSD basic network: inspired by the traditional SSD model design structure, the first 14 improved deep separable convolutional layers in the previously improved Mobilenet network are replaced with VGG16, which is used to improve the backbone network of the algorithm [29]. Then, add the feature extraction performance of the model to it; after the replacement of the basic network, add a convolutional layer with a decreasing correlation size to obtain deeper feature information of the image [30]. At the end of the network, the classification layer used to analyse the category and the nonmaximum suppression layer to filter the regression box are connected to replace the basic network [31]. After the implementation of the abovementioned improvement strategy for the traditional SSD, the improved SSD model is trained in the data-related training set, and the specific model is designed.

### 2.6. Case Analysis

In order to evaluate the improved algorithm of the paper, the following will compare the average accuracy and detection speed of the improved SSD algorithm, the general Mobilenet-SSD algorithm, and the improved Mobilenet-SSD algorithm. The precision is closely related to the accuracy rate, calculated as in equation (7):

(7) $$\begin{array}{c} \text{precision}=\frac{T_{p}}{T_{p}+F_{p}}. \end{array}$$

*T*_*p*_ is the number of positive samples in the prediction of positive samples, and *F*_*p*_ is the number of positive samples in the prediction of negative samples. The surveillance video in the teaching process of a university is sampled by the Open Source Computer Vision Library (Open CV) operation frame, and actions such as raising hands and writing are selected for preservation and processing. Finally, 800 images were obtained. Using the data enhancement method mentioned above, after the image data enhancement processing, the final 1600 images were obtained as the data set of this experiment. In the training set, 400 pieces were randomly selected for the various actions of raising hands, listening to lectures, playing with mobile phones, writing, and sleeping, and a total of 2,000 pieces were used as the training set for this experiment.

## 3. Results

### 3.1. The Recognition Performance of Different Algorithms

For the traditional SSD algorithm, the unoptimized Mobilenet-SSD algorithm, and the optimized Mobilenet-SSD algorithm, after the above training set is trained, the average accuracy and detection speed of each model in the data set are shown in Figure 9.

In Figure 9, after comparing the target recognition performance of different models, the optimized Mobilenet-SSD model has a higher average accuracy rate than the traditional SSD algorithm and the unoptimized Mobilenet-SSD algorithm, reaching 82.13%, and the detection speed is up to 23.5 fps (frames per second). Compared with the SSD model with high accuracy and slow detection speed, the overall performance of the Mobilenet-SSD model with fast detection speed and low accuracy is better.

### 3.2. Accuracy Test of Specific Behaviours of Different Models

Table 1 shows the five behavior detection results on SSD and optimized Mobilenet SSD models. The specific behaviors are:attending class, raising hands, playing mobile phones, writing, and sleeping. The specific values of the test results are shown in Table 1.

In Table 1, the optimized Mobilenet-SSD algorithm has a recognition accuracy of 88.31%, which is lower than that of the previous algorithm. The accuracy of mobile phone playing behaviour is 79.15%, which is an improvement compared with 78.74% of the SDD algorithm. The detection accuracy of the remaining hand-raising and writing behaviours has been improved to varying degrees. The accuracy of sleeping behaviour has a downward trend. The change trend of the five behaviour detection accuracy is shown in Figure 10.

Figure 10 shows that the optimized Mobilenet-SSD model has different behaviour detection accuracies in the classroom. Except that the behaviour of listening to lectures and sleeping is easily affected by the interference of occlusion, the other three actions have better action detection accuracy than the traditional SSD model. In writing behaviour detection, the optimized Mobilenet-SSD model has a detection accuracy of 81.11%, which is the biggest difference with traditional SSD. Combining the two experiments, the optimized Mobilenet-SSD model is compared with the traditional detection model in behaviour detection accuracy and detection speed. It can provide English teachers with better feedback on the students' listening status during the teaching process, thereby improving the English classroom teaching efficiency.

## 4. Conclusion

Under the influence of the scale of teaching, the efficiency of English teachers in classroom teaching has been greatly affected. In this case, the use of classroom monitoring resources combined with in-depth learning target detection provides research ideas for improving student teaching efficiency. With the expanding teaching scale, English teachers' classroom teaching behavior has a greater impact on the teaching efficiency. Based on this, the use of relevant monitoring resources in the classroom combined with target detection in deep learning provides a research idea for detecting students' learning status and improving students' teaching efficiency. Therefore, the paper optimizes the SSD target detection algorithm. Through the analysis of the algorithm, the algorithm is optimized and improved aiming at the defects of large amount of basic network parameters and poor small target detection. Using RMSProp's optimization algorithm, the convergence speed of the algorithm is optimized. Through the related experiments of student behaviour analysis, it is confirmed that the accuracy of small target recognition has been improved without changing the operation speed of the traditional algorithm. The accuracy of the algorithm objectively reflects the better overall performance of the designed algorithm. The disadvantage is limited by conditions, the sample data selected for the experiment is not particularly sufficient, and it may have a certain impact on the final experimental results. In the follow-up exploration, the experiment was carried out since finding more sufficient sample data. The performance of the algorithm is more deeply understood, modern technical support is provided for teachers to understand the learning status of students, and the efficiency of English classroom teaching is improved. The research content has far-reaching significance.

## Figures and Tables

**Figure 1:** Activation function calculation process.

**Figure 2:** CNN structure.

**Figure 3:** Connection form of CNN.

**Figure 4:** Face recognition process.

**Figure 5:** Image preprocessing method.

**Figure 6:** Behaviour recognition process.

**Figure 7:** SSD network structure.

**Figure 8:** The replacement process of the basic network.

**Figure 9:** Different model recognition performance.

**Figure 10:** Comparison of different behaviour detection accuracy (A: listening to lectures, B: playing with mobile phones, C: raising hands, D: writing, E: sleeping).

**Table 1:** Different algorithm behaviour detection accuracy rate.

Algorithm\behaviour	Attend class	Play cell phone	Raise hands	Writing	Sleep
SDD	88.53%	78.74%	85.27%	76.09%	86.66%
Optimization of Mobilenet-SSD	88.31%	79.15%	86.76%	81.12%	85.04%

## Data Availability

The data used to support the findings of this study are available from the corresponding author upon request.
